The article "Genome-wide association mapping of bread wheat genotypes for sustainable food security and yield potential under limited water conditions" was retracted in 2022. Reasons: duplicate publication; compromised peer review; a conflict of interest; concerns about the authorship.

# Genome-wide association mapping of bread wheat genotypes for sustainable food security and yield potential under limited water conditions

**DOI:** 10.1371/journal.pone.0263263

**Published:** 2022-03-31

**Authors:** Hafiz Ghulam Muhu-Din Ahmed, Yawen Zeng, Muhammad Iqbal, Muhammad Abdul Rehman Rashid, Humayun Raza, Aziz Ullah, Muhammad Ali, Muhammad Majid Yar, Adnan Noor Shah

**Affiliations:** 1 Department of Plant Breeding and Genetics, Faculty of Agriculture and Environment, The Islamia University of Bahawalpur, Bahawalpur, Pakistan; 2 Biotechnology and Germplasm Resources Institute, Yunnan Academy of Agricultural Sciences, Kunming, China; 3 Department of Bioinformatics and Biotechnology, Government College University Faisalabad, Faisalabad, Pakistan; 4 Department of Plant Breeding and Genetics, University of Sargodha, Sargodha, Pakistan; 5 Department of Environmental Sciences, Faculty of Agriculture and Environment, The Islamia University of Bahawalpur, Bahawalpur, Pakistan; 6 Department of Agricultural Engineering, Khwaja Fareed University of Engineering and Information Technology, Rahim Yar Khan, Punjab, Pakistan; Faculty of Agriculture (FoA), Sher-e-Kashmir University of Agricultural Sciences and Technology of Kashmir (SKUAST-K), Wadura Campus, INDIA

## Abstract

Determining the genetic basis of yield and water deficient tolerance in wheat is vital for wheat breeding programs. Herein, a genome-wide association study (GWAS) was performed for water deficient and yield-related attributes on wheat genotypes with high-density Illumina 90K Infinium SNP array. Major yield and drought-related attributes were phenotyped on a panel of Pakistani and foreign accessions grown in non-stressed and water deficient stressed environments during two crop cycles. Among all accessions, highly significant variations were shown in studied environments for examined characters. Water deficient conditions, reduced the wheat yield and had strong and positive correlation among relative water content and grain yield per plant. Population structure analyses based on 90,000 SNP data, classify the accessions into 4 sub-populations. Marker-trait association analyses (MTA) revealed that 134 significant SNPs were linked with yield and drought tolerance attributes. Pleotropic loci *RAC875_s117925_244* and *RAC875_c16333_340* located on chromosome 5A and 2A respectively, were significantly linked with relative water contents (RWC), cell membrane thermo-stability (CMT), grain per spike (GPS), spikelet per spike (SPS) and grain yield per plant (GYP). The markers *Ra_c58279_684*, *BobWhite_c23828_341* and *IAAV3414* located on chromosomes 2A, 6B and 7B respectively, showed pleotropic effects for RWC, GPS and GYP under both environments. The current experiment not only validated several MTAs reported in other studies but also discovered novel MTAs which significant under drought-stressed conditions. A total of 171 candidate genes were recognized that could be cloned and functionally characterized for the respective associated traits. For RWC and CMT, total 11 and 3 associated SNPs were mapped on coding DNA sequence (CDS) of the identified candidate genes. Isolation and characterization of the candidate genes herein mapped SNPs will be useful in discovering novel genes underpinning drought tolerance in bread wheat to fulfill the wheat demand and sustainable food security under limited water conditions.

## Introduction

Confirming sustainable wheat yield to meet the needs of growing population under continuous variation in climate is a major challenge for wheat scientists and growers. So, it needs more advancement against biotic and abiotic stress tolerance. As the population continues to grow, the demand for wheat is also increasing and it is predicted to be increase up to 40% by 2030. Therefore, there is an urgent need to increase wheat production to ensure sustainable food security [1]. Various limiting factors leading to the decline in wheat production include low quality wheat seed, late sowing, unapproved sowing practices, poor soil fertility, uneven fertilization, inappropriate weed control, biotic and abiotic stress [2]. Wheat crop rank first among other cereal crops due to its nutritional importance and high utilization rate. Rapid population growth and healthier lifestyles have prompted wheat breeders accept new challenges to produce new wheat genotypes with higher yield, good quality and resistance to biotic and a-biotic stresses [3].

Due to constraints such as drought, the actual yield of wheat has not reached its potential, primarily due to irregular pattern of rainfall. It was reported that yield losses in wheat are 17%- 70% due to a shortage of water. Water deficient environment is the main problem of wheat yield loss. Due to this problem, translocation efficiency of photosynthetic activity affected and ultimately the wheat grains weight and total yield decreased [4]. Another study reported that, the 50–90% yield reduction under water deficit conditions as compared to its potential in several regions of the world. The wheat plant undergoes a severe reaction to drought stress at tillering, jointing, booting, anthesis and grain filling stages. Tillering stage in wheat is a crucial phase in which plant produce tillers, spike’s primordia, spikelet and floret. Water deficient conditions in this stage can decrease total wheat yield by 46% [5].

Drought stress is a complex mechanism because it depends on several factors such as: species of crops, intensity of drought, drought duration, and plant growth stages [6]. To develop water deficient tolerant varieties, it is necessary to know the mechanisms and behavior of plants under water deficit environment. To survive, plants under drought condition can use more than one mechanism. In this regard there are 3 basic phenomena that plants can resist in drought stress. (1) escape mechanisms (2) tolerance mechanisms and (3) resistance mechanisms [7, 8]. In the first phenomena, plant completes its life cycle before the drought begins. In second phenomena, the plant competes parallel with drought stress, e.g., closing the stomata and/or reducing the transpiration rate. In the third phenomena, plant proceeds phases against drought stress by increasing the pigmentation of photosynthates and retain the ratio of root/shoot to efficiently partitioning the overall assimilate [8, 9]. Although progress has been made in improving wheat breeding under normal water conditions, but little progress has been made for water deficit conditions [10]. In the context of water shortage, the problem has become more prominent, with large differences in yield between productive areas and rain-fed agricultural areas [1]. Approaches to decrease this gap include the advancement of genetics for water deficient conditions by determining the causes of water deficient tolerance and subsequent introgression of genes for specific characters associated to cultivated wheat genotypes. Application of such approaches in breeding schemes are the time-efficient and cost-effective technique against water deficit conditions [11, 12].

Producing of maximum yielded and water deficit tolerant genotypes is difficult by numerous complications because yield and water deficit tolerance related genes are complex and polygenic in nature. Several methods were considered for selecting bread wheat varieties against water deficit environments. Previously wheat breeders [13] suggested that relative water contents related traits in wheat crop used as selection criteria for drought resistance. Almeselnani and other researcher [14] reported that this wheat trait is the best criterion for selecting drought-tolerant genotypes. The relative-water-contents (RWC) in terms of their relation to the volume of the cell can indicate the stability among the water uptake by the plants and expansion by transpiration [15]. An experiment was conducted by wheat researchers [16] in normal and water-deficit environments and they select the drought-tolerant varieties, which had optimum RWC in wheat. Selection of wheat genotypes based on these drought-related traits is informal, inexpensive, and less time-consuming. Various efforts have been made to increase wheat yield under drought stress using traditional breeding methods, but these strategies do not contribute more than 1% to the increase in annual yield [1, 17].

In coming days, the wheat breeding systems will depend upon discovering genetic and molecular potential of heat and drought tolerance using QTLs mapping, SNPs, association Mapping (AM) and next generation sequencing (NGS) studies. Genome-wide association mapping studies (GWAS) with genotypic and phenotypic data from association panels has been proved to be a robust method to detect quantitative trait loci (QTLs) linked with desired and target attributes [18]. In GWAS using of different set of germplasm which provide a wider range of genomic regions/allele frequencies at maximum resolution, without any bi-parental mapping population [19]. Genome wide association studies (GWAS) also explore the genetic mechanisms of attributes and their responsible genes. It is a useful technique with more accurate results because of having more genetic diversity and historically recombination of alleles between associated panels [4, 11]. It is useful to identify the genomic regions linked with drought tolerance and yield-related characters in various association mapping panels.

In the current experiment, a diverse panel of spring wheat accessions was genotyped with 90,000 SNPs array as well as phenotyped under normal and water deficit environment for two cropping cycles in 2017–18 and 2018–19. In this study, novel SNPs were found to be associated with key drought tolerance traits. The significantly associated SNPs with yield and water stress tolerance related indices were mapped on bread wheat reference sequence v1 and candidate genes were identified.

## Materials and methods

### Plant material

A panel of 96 Pakistani and foreign spring wheat accessions preserved at the department of Plant Breeding and Genetics, University of Agriculture Faisalabad, Pakistan (PBG-UAF) was used in this study. According to the maintained source, the 22 genotypes (G1 to G22) from advance breeding lines, established in PBG-UAF, while 26 genotypes (G23 to G46) from foreign source and the 48 genotypes G47 to G96 from locally cultivated Pakistani wheat varieties. The detail information about genotype code, origin, name and pedigree record is presented in S1 Table in S1 File. The association panel was sown in non-stressed and water deficient environments in the research area of PBG-UAF in triplicates fashion with a randomized complete block design of two consecutive harvesting activities in 2017–18 and 2018–19. In non-stressed experiment, irrigation were given at three critical stages; the first irrigation was applied at tillering stage (35 DAS (Days after sowing)), second irrigation was given at booting stage (85 DAS) while the third irrigation was given at milking stage (112 DAS) [20]. In the present study, water stress was used at tillering stage by missing the irrigation. Each genotype was sown in 1m long experimental unit with 3 replicates, maintaining P×P distance 15cm and R×R distance was 30cm. Only 2 seeds of each genotype were dibbled/hole and a healthy seedling was kept after germination by thinning. All other agronomic practices like fertilizer applications, hoeing, weeding, etc., were applied homogeneously to reduce the experimental error in both environments during both seasons.

### Phenotyping

At maturity, data were recorded from each of the ten plants of each replication for plant height (PH), numbers of tillers per plant (NTP), spikelet per spike (SPS), grain per spike (GPS) and grain yield per plant (GYP) under non-stressed and water deficient conditions for each year. Relatives water contents were measure by using the following formula [21]:

RWC(%)=[(FW‐DW)/(TW‐DW)]×100

Where, FW = Fresh Weight, DW = Dry Weight and TW = Turgid Weight.

Cell membrane thermo-stability (CMT) measured by using the previously described procedure [22]. Two fully developed leaves were taken from tagged wheat plants and each leaf was cut into two pieces, which were considered as normal and as heat-treated. Put halves of the leaves into two tubes having 10 ml of distilled water for 18h at 10°C. After washing the leaves, 15 ml distilled water was added. Then, put all the tubes in water bath while the one half of each test tube kept at 25°C and the other half at 45°C for 1hour. Both normal and heated leaves were further kept for 18h at 10°C to maintain the contents. The conductivity data were measured at 25°C with an electrical conductivity (EC) meter for control (C_1_) and heated (T_1_) tubes. The leaves were again heated for 1h. Another conductivity data of the aqueous phase (T_2_ and C_2_) was observed at 25°C after cooling the leaves. Cell membrane thermo-stability (CMT) was also expressed as percent relative injury (RI%) [22].

Cell membrane thermo-stability, CMT (%): [1- (T_1_/T_2_)] ×100
Relative Injury (RI) % = 100-[[1-(T_1_/T_2_)]/[1-(C_1_/C_2_)] ×100].

Where, C and T represent the electrical conductivity of normal and heated samples while the subscript 1 and 2 indicate electrical conductivity readings before and after autoclaved, respectively.

### Statistical analysis

Scored data were used for pooled analysis of variance (ANOVA) procedure using the GenStat^®^ Ver.17 [23] for studied attributes in non-stressed and water deficient environments. Pearson’s correlation coefficients (r) were measured to determine the correlation between yield and drought related characters using the SPSS ver.23 [24] in both environmental conditions. For ANOVA and correlation analysis significance of results were considered at α = 0.01 (highly significant) and α = 0.05 (significant outcomes) in this study.

### Genotyping of spring wheat genotypes

Each genotype was sown in polyethene bags and used the fresh leaf of 15-day wheat seedlings for DNA extraction according to the procedure of the CIMMYT Molecular Genetics Manual [25]. The DNA of each genotype (70–100 ng/μl) was stored in 96-well plates and sent to CapitalBio® at Beijing in China for genotyping using Illumina 90K Infinium high-density SNP array [26]. The genome-wide position of SNPs in terms of genetic distance (cM) located on chromosomes according to the consensus genetic map of bread wheat 2015 were used in current experiment [26]. During data analysis, monomorphic SNPs, missing values <20%, minor alleles and allelic frequency <5%, were excluded.

### Population structure and linkage disequilibrium (LD)

Bayesian clustering procedure was used with SNPs to categorize clusters of genetically similar genotypes through the statistical analysis STRUCTURE v.2.3 [27]. Burn-in iterations of 10^4^ cycles and admixture model selection was applied. An ad-hoc method based online tool “Structure Harvester v0.6.93” was practiced to attain high value or peak of ‘‘K” for authentication the STRUCTURE results [28]. We select the K value ranged from one to ten and six independent runs to achieve the reliable effects. Genome-wide linkage disequilibrium (LD) decay examination was attained by computing pairwise marker allele squared correlation (*r*^2^) and plotting the *r*^2^ value against the genetic distance (cM) using genome association and prediction integrated tool (GAPIT). This is an innovation in the R package, which provides some probability accuracy and calculation functions [12].

### GWAS analysis

GAPIT tool was practiced with modal selections preference to check the dependability of the results [29]. It implements unconventional statistical methods, including compressed mixed linear modal (CMLM) and CMLM-based genomics prediction selections, and determine the false discovery rate (FDR) [29, 30]. The threshold for describing a marker to be significant (p-values) was measured at 10^−3^ or above [18]. The significance level for *p* values were measured after Bonferroni adjustment (P = 1/n, n = total number of SNPs) [31]. To determine the relevance of the applied model for GWAS, quantile-quantile (QQ) plot was derived among the observed and expected log10(*P*) values [29]. To describe the unclear correlation obtained from population structures, covariate from STRUCTURE [27] were measured as fixed effects using the principal components through GAPIT [29, 32]. The mysterious associations among genotypes were estimated using a kinship matrix in the incorporated MLM [33]. Overall, 35,320 of the 81,000 functional iSelects beads chip analyses visually exhibited polymorphisms and detected on the publish genetics maps [26] in studied genotypes.

### Authenticating SNPs and recognisation of candidate genes

The wheat reference genome (IWGSC RefSeq v1.0) and gene annotations in GFF3 format were regained from the *Ensemblgenome* database (https://plants.ensembl.org/Triticum_aestivum/Info/Index) ftp://ftp.ensemblgenomes.org/pub/plants/release-44). The SNP sequence was aligned to wheat genome through blastn program with stringent E-values of 0.0001. For every SNP, only the best scoring hit was retained, and genomic position was annotated into 5’-UTR, 3’-UTR, CDS, intron, intergenic regions conferring the genomic regions offered in the GFF3 files. The intergenic regions were distinct as a genomic region with no annotated genes. The annotated genes within ±250Kb of the mapped SNP were considered as candidate as described in previous study [34].

## Results

### Phenotypic evaluation

In this study, analysis of variance (ANOVA) of 96 spring wheat accessions showed significant effects on phenotypic variation (P < 0.01). All traits showed significant effects among studied accessions as exhibited in S2 Table in S1 File. Descriptive statistics data of observed characters in non-stressed and water deficient environments based on average data over years have presented in S3 Table in S1 File. Broad-sense heritability of the studied indices was calculated and given in S2 Table in S1 File. The highest heritability was observed for NTP with the values of H^2^ = 83.41 and H^2^ = 77.23 under normal and drought conditions respectively. Average value of plant height was 97.67cm and 80.68cm under normal and water deficient environments, respectively. Relative water contents (RWC) and cell membrane thermostability (CMT) had mean values 76.11% and 66.20% under normal conditions while in drought conditions as 74.22% and 64.18%, respectively. Number of spikelet/spike and number of grain/spike exhibited mean performance as 18.87 and 47.40 under normal conditions, while, 10.90 and 32.00 under drought condition, respectively. Average value of grain yield per plant was 21.49g and 14.30g under non-stressed and stressed conditions, respectively. Plant height (PH) was negatively associated with all studied traits in non-stressed and water deficit conditions. The RWC was positively correlated with CMT, SPS, GPS and GYP under all studied environments. Water deficit tolerance related characters such as RWC and CMT were strongly and positively linked among themselves, while a negative correlation with plant height under both conditions was observed (Table 1). The yield related traits like SPS, GPS and GYP exhibited positive correlation with each other in non-stressed and water deficient conditions. GAPIT diagnosis phenotypic variation in drought and yield-related traits which including the scatter plot, histogram, box plot and accumulative distribution are mentioned in S1-S14 Figs in S1 File.

**Table 1:** Pearson’s correlation coefficient of studied attributes based on data averaged over years under normal and drought conditions.

Traits	Env.	PH	NTP	RWC	CMT	SPS	GPS
**NTP**	N	-0.22	** **	** **	** **	** **	** **
	D	0.26*		** **	** **	** **	** **
**RWC**	N	-0.31^*^	0.54^**^				
	D	-0.26^*^	0.55^**^				
**CMT**	N	-0.31^*^	0.43^**^	0.92^**^			
	D	-0.31^*^	0.46^**^	0.85^**^			
**SPS**	N	-0.15	0.35^**^	0.56^**^	0.56^**^		
	D	-0.27^*^	0.56^**^	0.91^**^	0.89^**^		
**GPS**	N	-0.31^*^	0.42^**^	0.88^**^	0.92^**^	0.56^**^	
	D	-0.30^*^	0.51^**^	0.85^**^	0.83^**^	0.88^**^	
**GYP**	N	-0.25^*^	0.54^**^	0.91^**^	0.93^**^	0.50^**^	0.91^**^
	D	-0.25^*^	0.51^**^	0.92^**^	0.86^**^	0.89^**^	0.84^**^

PH = Plant height, NTP = number of tillers per plant, RWC = Relative water content, CMT = Cell membrane thermo-stability, SPS = Spikelet per Spike, GPS = Grain per spike, GYP = grain yield per plant, SE = Standard error, N = normal, D = drought, Env = environment

* = Significant (α = 0.05) and

** = Highly significant (α = 0.01).

### Population structure

The results from the structure harvester displayed that the uppermost peak of K = 4 which depended on the rates of changes in the log probabilities of data among successive K-value (S15 Fig in S1 File) that was found on the second order derivation on the variance of the maximum probability of model to give a specific K. Delta K exhibits only the highest clustering level and number of subpopulations in main populations. Results from STRUCTURE analysis (S16 Fig in S1 File) exhibited that total 12 accessions (G1-G10, G27- G28) included in the first group. In the second group total 14 genotypes (G11-G22, G29-G30) were recorded. The third group included the total 39 genotypes from G34 to G72. Three genotypes from G31 to G33 exhibited mixed genetic material from above mentioned (second and third) groups. The fourth group contained total seventeen genotypes from G73 to G89. Total 6 accessions from G90 to G96 revealed the collective genetic material from the third and fourth group.

### Genome-wide marker trait associations for studied attributes

In this study, 35,320 high density SNP markers from the 90K Illumina iSelects SNP array were evaluated to perceive SNPs associated with water deficit tolerance and yield-related indices. Before analyses of GWAS and genomic prediction, scientists validated and maintained quality of genotypic data. The GAPIT provides a series of diagnostic tools to help users perform quality control on genotypes. These tools include histograms and accumulative distributions of marker density and decay plots of linkage disequilibrium over distance (LD). Linkage Disequilibrium (LD) among SNPs under study was presented in S46 and S47 Figs in S1 File. Linkage disequilibrium was measured as R square for pair wise markers and plotted against their distance. Marker-trait associations for these indices in non-stressed and water deficit environments examined. A total of 134 significant SNPs was correlated with observed characters, out of them 66 and 68 MTAs were scored in non-stressed and water deficit environments, respectively, at or above–log 10 (*P<* 0.0001) threshold level using MLM (mixed linear model) for seven yield and water deficit tolerance related traits (S4 and S5 Tables in S1 File). Manhattan plots (S17-S28 Figs in S1 File) presentation the site of significant SNPs at -log10(p) which significantly linked with the desired characters and examined environments. The Quantile-quantile (QQ) plot developed to verify the results of Manhattan plots as mentioned in the S29-S42 Figs in S1 File. A heat-map about the information mentioned in kinships matrix is developed (S43 Fig in S1 File). The 3D plot of first three PC of studied attributes mentioned in S44 in S1 File.

### Morphological attributes

Seven markers showed highly significant association with PH which found on chromosomes 2A, 4A, 6A, 7A and 6B in non-stressed condition (S17 Fig in S1 File). Associated loci of this trait showed phenotypic variation explained (PVE) from 12.91% to 16.03% of the total phenotypic variation (S4 Table in S1 File). Under water deficit condition, seventeen SNPs were strongly associated with PH on chromosome 1A, 3A, 4A and 5A, 7A, 2B and 3D (S18 Fig in S1 File). Total phenotypic variability by these associated markers range from 12.83% to 20.43% (S5 Table in S1 File). Number of tillers per plant (NTP) was highly linked with sixteen markers in non-stressed environment. Ten MTAs were detected on chromosomes 4A, two on 2A, two on 6A, one on 5A and one 1A (S19 Fig in S1 File) for this attribute. These sixteen NTP related markers explained the total phenotypic variation 14.04% to 17.97% (S4 Table in S1 File). Under drought condition, seven significant SNPs were strongly linked with NTP as well as four markers detected on chromosome 5A, 2 SNPs on chromosome 2A and one on 4A as mentioned in S20 Fig in S1 File. These markers explained 12.53% to 14.1% of the phenotypic variation in NTP under drought condition (S5 Table in S1 File).

### Drought related attributes

Under normal condition, relative water contents (RWC) was highly linked with seven markers. Two significant MTA associated with RWC were detected on chromosome 2A, 2 MTA on 5A, 2 on 7B and 1 on 6B as mentioned in S21 Fig in S1 File. These seven RWC related markers explained 16.54% to 19.91% of the variability in this attribute (S4 Table in S1 File). The marker (*wsnp_Ex_c5412_9564046*) explained the highest phenotypic variation (19.91%) on chromosome 2A at position 78.03 cM for this trait. Under drought condition, 10 significant SNPs were positively associated with RWC and situated on chromosomes 1A, 2A, 3A, 5B, 6B and7B (S22 Fig in S1 File). These markers explained 18.02% to 24.71% of the phenotypic variability in RWC under drought condition. The marker (*Excalibur_s112663_236*) located on chromosome 1A at 155.80cM distance exhibited highest phenotypic variability 24.71% in the current study. In non-stressed environment, the cell membrane thermo-stability (CMT) was highly correlated with eight MTAs, out of them, three MTAs were situated at chromosome 7B, two on 5A while one association on each of chromosomes 6A, 6B and 2A (S23 Fig in S1 File). These markers explained the phenotypic trait variability from 16.51% to 21.21% in the present study. Significant MTAs for CMT were distributed on all wheat genomes, including four SNPs from B-genome, three from A-genome and one from D-genome (S4 Table in S1 File). The marker (*RAC875_s117925_244*) showed more phenotypic variability (21.21%) on chromosome 5A at the position of 15.53cM under normal condition. Under drought-stressed condition, 12 significantly associated SNPs explaining phenotypic variability ranged from 17.83% to 23.09% in this attribute. Four SNPs were detected at chromosome 4A, two at each of 2A, 1B, 3B and 4B (S24 Fig in S1 File).

### Yield and yield related attributes

Total five significantly associated SNPs were recorded in current experiment for spikelet per spike (SPS) in non-stressed condition. Three SNP markers were identified at chromosomes 5A, one at each of 3A and 6D (S25 Fig in S1 File). For this attribute, phenotypic variations described by these SNPs marker fluctuated from 19.79% to 25.16% for this attribute. Under drought condition, ten significantly associated SNPs were positively linked with SPS. Out of them, two were situated at each of chromosomes 3A, 4A, 2B while the others on 2A, 7A, 1B, 4B, 6B (S26 Fig in S1 File). These SNPs had 14.05% to 24.59% variation in SPS under drought condition.

Fifteen markers were highly associated with grain per spike (GPS) in non-stressed environment which were found at chromosomes 2A, 5A, 7B and 6D (S27 Fig in S1 File). These significantly associated markers explained 16.62% to 21.54% of the variability in this attribute. Significant MTAs for GPS were dispersed on all three genomes, including, six SNPs on A-genome, seven at B-genome and two at D-genome (S4 Table in S1 File). Four significant markers were perceived for GPS under drought-stressed conditions. One marker was located on each of chromosome 1A, 4A, 5B and 7D explaining 14.43% to 16.66% variation for GPS under drought condition (S5 Table in S1 File). In non-stressed conditions, grain yield per plant (GYP) was positively correlated with eight SNPs. Out of them, three SNPs were found from chromosome 2A, 2 from 5A, 1from 6B and 2 from 7B (Fig 1). All these SNPs explained 15.95% to 19.04% of the phenotypic trait variability. Significant MTAs for this attribute was distributed across two genomes, including, five SNPs from A-genome and three from B-genome. The marker (*BobWhite_c23828_341*) explained more trait phenotypic variability (19.04%) at chromosome 6B with position 43.94cM while the marker (*Kukri_c55051_414*) from chromosome 5A with the position13.62 cM explained least variability (15.95%) in non-stressed environments (S4 Table in S1 File). Under water deficient environment, eight MTAs were observed to be significantly correlated. Out of them, two MTAs were detected from chromosome 1B, two from 4A and other from 1A, 3A, 7B and 5D (Fig 2). These significant MTAs explained trait phenotypic variability ranged from 16.06% to 23.88% under water deficient environment. These MTAs were distributed on all wheat genomes, including, four MTAs at A-genomes, three at B-genomes and one at D-genomes (S5 Table in S1 File).

**Fig 1:** Manhattan plots showing the location of significant SNPs and -log10(p) associated with grain yield per plant under normal conditions. The *blue horizontal line* designates the threshold of significance.

**Fig 2:** Manhattan plots showing the location of significant SNPs and -log10(p) associated with grain yield per plant under drought conditions. The *blue horizontal line* designates the threshold of significance.

### Genome-wide multiple traits loci associations

In genome A the markers (*RAC875_rep_c73318_362* and *RAC875_rep_c109969_119*) showed the least phenotypic variability 12.90% and 12.82% on chromosomes 6A and 5A having the position of 71.72 cM and 92.86 cM were considerably linked with plant height in non-stress and water deficient environments, respectively. Highest phenotypic variability 21.54% and 24.71% occurred in A genome represented by the significant SNPs *wsnp_Ex_c5412_9564046* and *Excalibur_s112663_236* from chromosomes 2A and 1A having the position of 78.03cM and 155.80cM were associate with GPS and RWC in non-stressed and water deficient environments, respectively. The significant markers, namely *wsnp_Ku_c43368_50890819* and *TA005830-0667* were correlated with PH in B genome from chromosome 6B (87.90cM) and 2B (110.82cM) explained 13.12% and 13.56% variation in non-stress and water deficient environment, respectively. In genome B the significant SNPs (*BobWhite_c23828_341* and *D_F5MV3MU01CCU25_62*) observed the maximum traits variation 19.04% and 21.66% from chromosomes 6B and 4B with the position of 43.94cM and 64.03cM for GYP and CMT in studied environments. The significant SNPs namely, *Kukri_c55362_75* and *Excalibur_c15009_2039* located on chromosomes 6D (18.99cM) and 3D (134.98cM) were associated with SPS and RWC in D genome showing more phenotypic variability 25.16% and 19.79%, respectively in the examined environments. The lowest phenotypic variation 16.51% and 13.74% existed in genome D depicted by the markers *RAC875_c16333_340* and *Kukri_c63797_354* on chromosomes 6D and 3D with the position 127.65cM and 142.31 cM were linked with CMT and PH in normal and water deficit environment conditions, respectively. Under water deficient condition, a pleiotropic locus (*RAC875_c16333_340*) for RWC and SPS was identified on chromosome 2A at the position 127.65 cM. The studied characters governed by a pleiotropic locus (*Tdurum_contig62744_393*) were associated with GYP and CMT on chromosome 4A at 154.30cM under drought condition as shown in S5 Table in S1 File.

### Authentication of SNPs and recognisation of candidate genes

Out of 93 SNPs which were observed to be linked with various traits under study, 80 were effectively mapped on the bread wheat reference sequence. The chromosome number, strand and genomic position, of each mapped SNP have been given in S6 Table in S1 File. The SNPs mapped in coding DNA sequence, introns and3’UTR (3’ untranslated region), extended ±250Kb and inter-genic region were 26, 5, 8, 39 and 2, respectively (S45 Fig in S1 File). To validate MTAs, candidate genes were recognized surrounding ±250Kb of the mapped SNPs. Total 171 candidate genes (S6 Table in S1 File) were identified for the 80 SNPs associated with studied traits and mapped on bread wheat reference sequence IWGSC RefSeq v1.0.

## Discussions

### Phenotypic evaluation

In this study, highly significant differences were observed among genotypes and environmental conditions, which showed the occurrence of variation and environmental effects on genotype performance in all studied traits as exhibited in S2 Table in S1 File [4, 11]. Heritability estimates provided the information about extent of which a specific genetic character to be transmitted to the successive generations. In current experiments, High heritability was reported in the studied traits under normal conditions, like NTP (83.41), followed by RWC (67.58), SPS (67.30) and GPS (63.22) which indicated (S2 Table in S1 File) that these were simply inherited traits and most likely the heritability was due to additive gene effects and selection may be effective in early generations for these traits. Previous studies have also reported the high heritability in GPS and GYP as complex traits. Average value of grain yield per plant was 21.49g and 14.30g under non-stressed and stressed conditions, respectively. Adverse possessions of water deficient stress on wheat performance in addition to genotypic variation in response to drought have already been observed [8]. It is also reported that in wheat crop maximum loss of grain development due to water deficient conditions at anthesis and post-anthesis stage [35] ultimately reduce overall grain yield per plant [36]. The occurrence of water deficiency at booting stage directly reduced the number of spikelet per spike, which ultimately reduced the number of grains per spike and grain yield per plan. The findings agreed with our results regarding water deficient stress at the booting stage. Few motives are associated with the limit of physiological and biochemical pathways due to water shortage, which caused yield losses in wheat [7, 8]. Plant height (PH) was negatively associated with all studied traits in non-stressed and water deficient environments as previous study supported our findings [37], which showed that no association was established with other observed parameters. As a result, the selection for plant height is not a favorable criterion for these genotypes. The yield related traits like SPS, GPS and GYP showed positive association with each other in non-stressed and water deficient environments and the selection of mentioned traits will be fruitful for this germplasm [20, 38]. Cell membrane-thermo stability (CMS) and Relative water content already used to select tolerant varieties [39]. The mean variability of drought and yield related traits was observed. Among the genotypes with variable performance in water deficient environments, the best performers were categorized as drought tolerant genotypes. Based on these evidences the tolerant genotypes G6 followed by G1 and G21 as shown in Table 2.

**Table 2:** Best performance wheat genotypes under both conditions on data averaged over years.

Trait	Normal	Drought
PH	G89 followed by G77, G82, G91 and G96	G89 followed by G77, G82, G91 and G96
NTP	G21 followed by G6, G16, G39 and G1	G 39followed by G6, G1, G16 and G21
RWC	G6 followed by G21, G16, G39 and G1	G6 followed by G39, G16, G21 and G1
CMT	G6 followed by G21, G16, G39 and G1	G6 followed by G21, G16, G39 and G1
SPS	G6 followed by G39, G6, G21 and G1	G6 followed by G21, G16, G39 and G1
GPS	G21 followed by G6, G1, G39 and G16	G6 followed by G21, G16, G39 and G1
GYP	G1 followed by G11, G6, G16 and G21	G1 followed by G11, G6, G21 and G16

PH = Plant height, NTP = number of tillers per plant, RWC = Relative water content, CMT = Cell membrane thermo-stability, SPS = Spikelet per Spike, GPS = Grain per spike, GYP = grain yield per plant, SE = Standard error, N = normal, D = drought, G = genotype.

### Population structure

The Bayesian approach made in statistical software packages STRUCTURE versions 2.3.3 used to assess the genetic structures of 96 bread wheat genotypes. The observed accessions were classified into 4 sub-group based on molecular data. Various kinds of colors in S16 Fig in S1 File show the discrete groups and overall studied genotypes assigned into 4 sub-groups. This practice previously also used in wheat breeding program by several experts and were attained the descriptive results [1]. STRUCTURE analysis recommended that 96 genotypes originated from diverse progenies. However, the known origin indication according to preserver of 96 wheat genotypes and pedigree records, exhibited three types of population but genetically these genotypes were divided into four sub populations. According to the maintained sources (S1 Table in S1 File), the first group consisted of the accessions G1 to G22 from advance-breeding lines, established in PBG-UAF, while second group had accessions G23 to G46 from foreign source and third group had the accessions G47 to G96 from locally cultivated Pakistani wheat varieties. In wheat breeding program these practices also used by several wheat breeders [11, 12]. STRUCTURE analysis recommended the divergences among 96 bread wheat genotypes which represented the genetic resemblance within groups and genetic differences between the groups. Mainly, outcomes were practically deliberating to the already identified pedigree record and origin of wheat accessions. Determination of genetic diversity would be helpful to recognize the diverse accessions for the improvement and progress the future wheat breeding program [34]. Those accessions having diverse genetic makeup can be designated for required combinations to produce multiple and significant traits to gain a better yield. Discernment of wheat accessions based on their genetic basis will be beneficial for effective and early screening of anticipated accessions in wheat breeding program for producing high-yielded wheat varieties.

### Genome-wide marker traits associations

Genes and QTLs related to water deficit tolerance and yield characters in whole wheat genomes, were distributed across 21 chromosomes described by several wheat breeders [40, 41]. Marker-trait association (MTA) study recognized the connection between a particular morphological and genetic variation within a genome, which ultimately perceived locus underpinning related characters at the end [42]. In this study, 35,320 high density, polymorphic SNP markers from 90K Illumina iSelects SNPs array [26] were examined to notice SNPs associated with drought and yield associated indices. The density of SNPs under study is precarious to develop. The denser SNPs showed the best genome coverage, which were detected by the comparison among the studied SNPs density and the LD decay. Marker-trait associations (MTA) for these characters in non-stressed and water deficient environments were detected. The *blue horizontal line* on Manhattan plot entitles the threshold level (*P<* 0.0001) of significance for SNPs with specific traits. The quantile-quantile (QQ) plot between the detected negative base 10 log of the *P*-value and expected negative base 10 log of the *P-*value with the assumptions that the *P*-value monitor a constant [0,1] scattering was observed as well. The dotted line showed the 95% confidence intervals for the QQ-plots in the null hypothesis of zero (0) correlation among SNPs and the studied traits. The kinships matrix helped in GWAS was envisioned by heat-map. To shrink computational problems, heat-map is not created when the sample size increased to 1000. The 3D plot of the first three PC categorized the association panel in four groups with high diversity within groups as was reflected from results of population structure analysis.

MTAs for PH were dispersed on overall seven (07) chromosomes, eight MTA at A-genomes, six at B-genomes and three at D-genomes under drought-stress condition. Earlier researches had reported MTAs for PH [41] and stated that, two SNPs situated at chromosomes 1A and 2D are linked with plant height under water deficit conditions. The QTL region on 6A for PH was < 10 cM far at the long arm and linked with GPS and GYP (S5 Table in S1 File) [43]. Similar results of plant height in accordance with the current study were described to be linked with genomic parts from chromosomes 1B [44], 2B, 6A [45], 5A, 5B and 6B [46]. In this experiment, MTA for NTP were dispersed across the A genome under water deficit conditions. Wheat scientists [12] found the significant SNPs on 5A for this trait under water deficient environment. MTAs for RWC were dispersed across 10 chromosomes with five SNPs at A-genomes, 3 at B-genomes and 2 at D-genomes (S5 Table in S1 File). The 5 QTL for RWC in wheat crop were reported on chromosome 1B-1D-2B-6A and 7B by many wheat scientists [47]. The significant MTAs for CMT were distributed across A and B genomes, including 6 SNPs at A-genome and 6 at B-genome. Thomelin et al [48] evaluated a water deficit and high temperature tolerant QTL *qDHY*.*3BL* in ~ 1Mbp on chromosomes 3B, having twenty-two responsible genes for CMT. In this trait, 20 SNPs were reported, which showed a significant association [39]. These were situated at chromosomes 1A, 1B, 2A, 3A, 4A, 4B, 6B and 7B and similar with our findings. Significant MTA for SPS were distributed across 2 genomes including 6 SNPs on A-genome and four on B-genome. Wheat scientists [41] reported that in water deficit conditions, spikelet per spike was significantly linked with 8 SNPs situated at chromosomes 1B, 2B, 4B, 6B, 2D and 5D, whether in similar condition, 7 significantly markers traits association were reported which is situated at chromosomes 5A, 1B, 4B, 5B, 6B and 2D. Three SNPs associated with SPS located on chromosome 2A, 2B, 7B were reported [41] which supports our results for this study.

Highly phenotypic attributes associations can be described in relation to directly or indirectly influence one attribute to other attributes. Within the genome, these attributes could be controlled by pleiotropic loci. It is proved by the presence of numerous MTAs in which one gene will show the pleiotropic influence on more associated attributes [49]. MTA for GPS were dispersed across 3 genomes; two at A-genomes, one at B-genomes and one at D-genomes under drought condition (S28 Fig in S1 File). Remarkably, chromosome 5B stated by wheat scientists [43] that harbor a region regulating numerous yield-related attributes was identified which have genomic parts linked with spikelet per spike and GPS in current experiment. The record noteworthy and steady QTL responsible GPS was observed on chromosome 1A and 2A commonly found across different environmental conditions [50]. MTA controlling GYP were found on chromosomes 1A, 4B, 6B, and 7D [11]. Earlier detected MTAs for GYP in wheat crop were at chromosome 1B [44], 2B [51], 3A [6], 7A, 7B and 3D [52], 5B [53].

The marker locus on 5A was correlated with GYP in normal condition described previously [12]. Similarly, Edae et al. [43] described significant MTAs for GYP at chromosome 4A, 1B, 5B, and 2B. Moreover, Lozada et al. [54] also specified MTAs for this trait on chromosomes 5A, 1B, 2B and 4B [18] identified MTA for GY from chromosome 5A. Lopes et al. [55] recognized MTA for GYP on 2D, and [19] informed GYP linked MTAs on 1B. Pinto et al. [44] also noticed GYP linked MTA on 4A which described 27% of variations in water deficient environments. MTAs for GYP were recognized in the present study were precise to different environmental conditions suggesting dynamic nature of genetics corresponding to the grain yield per plant (GYP) [54]. The highest number of marker-trait associated genome region and chromosomes are mentioned trait-wise in Table 5.

### Genome-wide multiple traits loci associations

Multi-trait-loci were seemed on chromosome 2A (PH, NTP, RWC, GPS and GYP), 5A (NTP, RWC, CMT, SPS, GPS and GYP), 6B (PH, CMT, GYP, GPS and RWC), 6D (CMT, SPS and GPS), 7A (PH and CMT) and 7B (CMT, RWC, GPS and GYP) under normal condition. The *Q* gene situated at chromosome 5A confirmed the easily threshing of spikes, pleiotropic effects and several domestically associated attributes like plant height, spike length and emergence time of spike [56]. *TaTEF-7A* and *TaMOCI-7A* also have reported as linked with SPS and located on chromosome 7A [57]. Multi-trait loci were identified on chromosomes 1A (PH, RWC, GPS and GYP), 1B (CMT, SPS, GYP), 2A (NTP, RWC, CMT and SPS), 2B (PH and SPS), 3A (PH, SPS, RWC and GYP), 3D (PH and RWC), 4A (PH, NTP, CMT, SPS, GPS and GYP), 4B (CMT and SPS), 5B (GPS and RWC), 7A (SPS and PH) and 7B (RWC and GYP) under drought-stressed conditions (Table 3). The distal areas of chromosomes 7A and 7B are described to comprise QTL for yellow pigment content of grain, which directed by *Phytoene synthase*1 (PSY-1) genes, the occurrence of these genes can effect for the pleiotropic link at 7B [58]. The *TaSnRK2* gene determined sucrose non-fermenting 1-related protein kinase situated at chromosomes 4A and 4B. Its role is important for responding against several environmental conditions and depict significant association with SPS and GPS [18, 59, 60]. Wheat yield related genes, such as *TaGW2-A1* at 6A *TaTGW6-A1* at 3A, *TaCwi* at 2A, *TaGS5-A1/TaGS-D1* at 4A, *TaSus1* at 7A and *TaSus2* at 7B reported by wheat scientists [40, 61, 62].

**Table 3:** Highest number of significant MTAs.

Significant MTAs					
Genome and Chromosome Wide			Traits wise		
Genome	Normal	Drought	Traits	Normal	Drought
A Genome	Total 43 MTAs (1A = 1, 2A = 13,5A = 11,6A = 4,7A = 2,3A = 1,4A = 11)	Total 38 MTAs (4A = 11, 3A = 8,2A = 7,1A = 4,5A = 6, 7A = 2)	PH	7	17
			NTP	16	7
B Genome	Total 19 MTAs (7B = 13, 6B = 6)	Total 23 MTAs (2B = 8, 1B = 5,3B = 2,5B = 2,7B = 2, 6B = 1)	RWC	8	10
			CMT	8	12
D genome	Total 4 MTAs (6D = 4)	Total 7 MTAs (3D = 4,1D = 1,5D = 1,7D = 1)	SPS	5	10
			GPS	8	4
			GYP	15	8

MTAs = Markers Traits Associations, PH = Plant height, NTP = number of tillers per plant, RWC = Relative water content, CMT = Cell membrane thermo-stability, SPS = Spikelet per Spike, GPS = Grain per spike, GYP = grain yield per plant.

A pleiotropic locus is correlated and alters the appearance of several phenotypic attributes. In the current experiment, many pleiotropic loci were recorded, under normal conditions, pleiotropic locus (*RAC875_s117925_244*) on chromosome 5A at 15.53 cM were significantly linked with yield and drought-related traits such as RWC, CMT, GPS and GYP. Another pleiotropic locus (*wsnp_Ex_c5412_9564046*) at chromosome 2A on the positions 78.03cM was also linked with RWC, GPS and GYP. The examined characters like RWC, GPS and GYP were influenced by a pleiotropic locus (*Ra_c58279_684*) on chromosome 2A at 78.03cM under normal conditions. The markers *BobWhite_c23828_341* and *IAAV3414* on chromosomes 6B and 7B at 43.94cM and 72.74cM, respectively, showed pleiotropic effects for RWC GPS and GYP as shown in S4 Table in S1 File. In this experiment, multi trait loci for yield and drought related characters were recognized on chromosome 2A, 5A, 7A, 6B and 7B in both environments as mentioned in Table 3.

### Authenticatiion of SNPs and recognisation of candidate genes

To authenticate the SNPs stated by Wang et al [26], the sequences of the SNP loci were mapped on currently available bread wheat reference sequence (IWGSC RefSeq v1.0). The candidate genes which could be cloned and functionally characterized for the mentioned associated trait were recognized. For relative water content (RWC) alone, which is a key trait for drought tolerance, 38 candidate genes were identified. Notably, 11 SNPs linked with RWC were mapped in CDS of the respective candidate genes (S6 Table in S1 File). For Cell Membrane Thermo-stability (CMT), 3 SNPs were mapped in CDS of corresponding candidate genes. For grain yield related traits 15 SNPs were mapped in CDS. For GYP, fourteen and twenty-one candidate genes were recognized in non-stressed and water deficient environments, respectively. The candidate genes stated here in current experiment were more diverse than those which have been cloned so far, such as *TaSnRK2*.*10-4A*, *TaTGW6-A1*, *TaFlo2-A1*, *TaGS53A*, *TaGASR7-A1*, *TaSAP1-A1*, *TaCwi-A1*, *TaGW2*, *TaGS1a* and *TaGS-D1* [60, 61, 63]. Cloning and characterization of the candidate genes in which SNPs were mapped in CDS would more likely result in discovering novel genes underpinning yield potential and drought tolerance in bread wheat.

## Conclusion

Drought stress reduced grain yield and strong positive correlation exist among yield and drought related attributes like RWC and CMT with grain yield per plant. Therefore, selection based on these traits would be fruitful. The parameter like plant height that was negatively associated can affect the performances of other attributes during selection procedures. In this experiment, numerous pleiotropic loci were known, under normal conditions, pleotropic locus (*RAC875_s117925_244* and *wsnp_Ex_c5412_9564046*) on chromosome 5A, 2A were significantly associated with yield and drought tolerance linked characters like RWC, CMT, GPS and GYP. The Markers *BobWhite_c23828_341* and *IAAV3414* on chromosomes 6B and 7B showed pleiotropic effects for RWC GPS and GYP. Under drought condition, pleiotropic locus (*RAC875_c16333_340* and *Tdurum_contig62744_393*) for RWC, CMT, SPS and GYP was identified on chromosome 2A and 4A. In this experiment, multi trait loci for yield and drought tolerance linked attributes was recognized on chromosome 2A, 5A, 7A, 6B and 7B under both environments. Furthermore, the predicted candidate genes wherein traits associated SNP markers were mapped in CDS could be functional genes for the respective yield and drought tolerance trait.

## Supporting information

S1 File Supplementary tables and figures. (DOC)
